The article "Harnessing the power of AI: Advanced deep learning models optimization for accurate SARS-CoV-2 forecasting" was retracted in 2025. Reasons: duplicated images; duplicated data; overlap with earlier publications; concerns about the data.

# Harnessing the power of AI: Advanced deep learning models optimization for accurate SARS-CoV-2 forecasting

**DOI:** 10.1371/journal.pone.0287755

**Published:** 2023-07-20

**Authors:** Muhammad Usman Tariq, Shuhaida Binti Ismail, Muhammad Babar, Ashir Ahmad

**Affiliations:** 1 Abu Dhabi University, Abu Dhabi, United Arab Emirates; 2 Universiti Tun Hussein Onn Malaysia (UTHM), Parit Raja, Malaysia; 3 Robotics and Internet of Things Lab, Prince Sultan University, Riyadh, Saudi Arabia; 4 College of Computer and Information Sciences, Prince Sultan University, Riyadh, Saudi Arabia; 5 Swinburne University of Technology, Melbourne, Australia; Huazhong University of Science and Technology, CHINA

## Abstract

The pandemic has significantly affected many countries including the USA, UK, Asia, the Middle East and Africa region, and many other countries. Similarly, it has substantially affected Malaysia, making it crucial to develop efficient and precise forecasting tools for guiding public health policies and approaches. Our study is based on advanced deep-learning models to predict the SARS-CoV-2 cases. We evaluate the performance of Long Short-Term Memory (LSTM), Bi-directional LSTM, Convolutional Neural Networks (CNN), CNN-LSTM, Multilayer Perceptron, Gated Recurrent Unit (GRU), and Recurrent Neural Networks (RNN). We trained these models and assessed them using a detailed dataset of confirmed cases, demographic data, and pertinent socio-economic factors. Our research aims to determine the most reliable and accurate model for forecasting SARS-CoV-2 cases in the region. We were able to test and optimize deep learning models to predict cases, with each model displaying diverse levels of accuracy and precision. A comprehensive evaluation of the models’ performance discloses the most appropriate architecture for Malaysia’s specific situation. This study supports ongoing efforts to combat the pandemic by offering valuable insights into the application of sophisticated deep-learning models for precise and timely SARS-CoV-2 case predictions. The findings hold considerable implications for public health decision-making, empowering authorities to create targeted and data-driven interventions to limit the virus’s spread and minimize its effects on Malaysia’s population.

## 1. Introduction

Malaysia has encountered significant obstacles in containing the virus’s proliferation and addressing its repercussions. Precise forecasting of the pandemic’s dynamics is essential for effective decision-making and resource distribution by healthcare institutions, governments, and policymakers. Recently, deep learning models have shown exceptional performance in tackling various challenges in healthcare, image processing, text recognition, and natural language processing. These models have been successfully employed for numerous SARS-CoV-2 predicting tasks, making their use for predicting the pandemic’s development in Malaysia particularly relevant.

In Malaysia’s context, multiple studies have used deep learning models for predicting the pandemic’s progression, but a few have used deep learning and optimization together in a single paper. The current paper has extended the deep learning models up to six models with an extended comparison of optimized and non-optimized algorithms. Further, most of the researchers have used only one to three models only. For instance, [1] utilized a multi-input multi-output CNN model to forecast SARS-COV-2 cases in several countries, including Malaysia. Their findings suggested that the CNN model effectively identified local patterns in the data and produced accurate forecasts. Likewise, other research such as [2] explored the use of LSTM and Bi-LSTM models for SARS-COV-2 forecasting in the region, showcasing their capacity to grasp complex temporal dependencies in the data and deliver dependable predictions. [3] used a hybrid deep learning model, SSA, and ConvLSTm network for predicting the wind speed. [4] used advanced comparative prediction models based on random forest, LSTM, and MLP that had high prediction accuracy for commodity prices using text mining methods. The deep learning models discussed in this review encompass Long Short-Term Memory (LSTM), Short-Term Memory (LSTM), Bidirectional LSTM (Bi-LSTM), Convolutional Neural Networks (CNN), CNN-LSTM, Gated Recurrent Unit (GRU), Recurrent Neural Network (RNN), and Multi-Layer Perceptron’s (MLP). These models have been used in various research projects to forecast SARS-COV-2 cases, fatalities, and recoveries, as well as to predict the effects of distinct government interventions and public health measures [5, 6].

### 1.1 SARS-COV-2 pandemic in Malaysia

Following the initial reported case in January 2020, Malaysia has enforced rigorous measures to manage the virus’s dissemination. The nation’s response has developed over time, adjusting to the pandemic’s shifting landscape. Key aspects of Malaysia’s response include lockdowns, travel restrictions, mass vaccination drives, healthcare infrastructure enhancement, and testing and tracing capabilities.

### 1.2 Model selection and evaluation

Choosing suitable models and evaluation methods for SARS-COV-2 forecasting can be daunting, considering the pandemic’s intricate nature and the various factors influencing its transmission. Researchers need to contemplate several aspects, such as model intricacy, interpretability, and generalizability when creating and evaluating forecasting models. Furthermore, the rapidly changing dynamics of the pandemic demand continuous model adaptation and assessment, as models that excel at one point may become less precise as the situation progresses. Despite these challenges, advanced deep-learning models have demonstrated the potential in capturing complex data patterns and providing accurate forecasts. By comprehending the challenges and complexities of SARS-COV-2 forecasting, researchers can persist in developing and refining models, ultimately contributing to informed policymaking, strategic resource allocation, and efficient public health interventions in Malaysia. Brief Comparative Studies in Malaysia Numerous studies have carried out comparative analyses of deep learning models to assess their performance in predicting pandemic cases in Malaysia.

[7–9] performed an extensive comparison of GRU, LSTM, and CNN models for forecasting cases in Malaysia. The authors utilized daily recoveries, confirmed cases, and deaths as input features for models and assessed their performance using metrics such as MAE and RMSE. The study aimed to identify the best deep learning model to capture complex temporal patterns in the data and provide accurate forecasts. The results revealed that both LSTM and GRU surpassed the CNN model in terms of prediction accuracy. [10–15]; used LSTM, GRU, and Transformer models for predicting SARS-COV-2 cases in Malaysia. They employed similar features as previous researchers, focusing on daily cases, deaths, and confirmed cases. Evaluation metrics such as MAE, RMSE, and MAPE were used. The study aimed to determine the best deep learning model for identifying the complex nature of the relationship between different features. The authors credited this finding to the Transformer model’s self-attention mechanism, which allowed it to capture complex dependencies in the data more effectively than the LSTM and GRU models. Furthermore, the Transformer model demonstrated faster training times and better scalability compared to the other models, making it a more practical choice for large-scale SARS-COV-2 forecasting tasks in Malaysia.

[16–21] used LSTM, GRU, and CNN-based models for predicting cases in Malaysia and various other countries. The authors employed daily confirmed cases as input features and evaluated the models’ performance using MAE and RMSE. Their study concluded that LSTM and GRU models outperformed CNN models, emphasizing the importance of selecting appropriate deep-learning models for pandemic evolution prediction in Malaysia. Researchers [22–25] compared LSTM, GRU, and 1D-CNN models in the context of forecasting future cases in Malaysia. They utilized similar features and evaluation metrics as earlier studies. The results revealed that GRU models exhibited the best overall performance, showcasing their potential for predicting cases in Malaysia. [26–30] provided a comparison of LSTM, GRU, and CNN models, employing features and evaluation metrics like MAE and RMSE, consistent with previous research. The importance of selecting suitable deep-learning models for case prediction was emphasized. In a comparison of LSTM, GRU, and Prophet models for forecasting cases in Malaysia [31–35], MAE and RMSE were used as evaluation metrics. The study found that LSTM and GRU models outperformed the Prophet model. [36–40] used LSTM, GRU, and 1D-CNN models, using daily confirmed cases, recoveries, and deaths as input features, and MAE, RMSE, and MAPE for evaluating model performance. The GRU model performed the best in this context. [41–43] conducted a comparative study on LSTM, GRU, and CNN models for Malaysia, using similar features and metrics as previous research (MAE and RMSE). The GRU model was found to achieve the highest prediction accuracy. [44–47] used LSTM, GRU, and CNN models, using MAE, RMSE, and MAPE alongside similar features as earlier studies. The LSTM model provided the best performance. [48–52] carried out a comparative study involving LSTM, GRU, and 1D-CNN models for Malaysia, using similar features and evaluation metrics as previous researchers. The LSTM model achieved the highest prediction accuracy in this context. [53] used the VMD-Staked GRU model to accurately predict individual stock finances from the industry environment factors that provide significantly improved predictions. [54] compared LSTM and other popular models for energy consumption forecasting that provided to have high accuracy for energy systems. [55] provided a comprehensive analysis using machine learning approaches that highlighted the rapid growth, geo trends, and their applications in various domains.

These comparative studies emphasize the significance of choosing the most appropriate deep-learning model for understanding the pandemic’s progression in Malaysia. While LSTM and GRU models have proven successful in capturing long-range dependencies in time series data, CNN models have also demonstrated effectiveness in certain scenarios. The selection of a deep-learning model should be based on the specific needs and limitations of the forecasting task, as well as the available data and computational resources. Moreover, these studies underscore the importance of employing deep learning models to generate accurate and dependable forecasts, which can aid decision-makers and public health officials in mitigating the pandemic’s impact in Malaysia.

## 2. Material and methods

We have focused on first performing different steps on the collected data and then performing tests using each deep learning model. Further, we have improved the models with Bayesian optimization to find out the difference between the optimization and without optimization of models. The study comprises data collection and preprocessing, model selection, model training and evaluation, and performance comparison.

### 2.1 Data collection

The study utilized daily SARS-COV-2 data from Malaysia, including confirmed cases, recoveries, and deaths. Data were gathered from official sources like the World Health Organization (WHO) and the Malaysia Ministry of Health. Additional data, such as government interventions, mobility patterns, and vaccination rates, were also collected to offer contextual information and enhance the models’ forecasting accuracy. The data chosen for this study was up until December 2022. Fig 1 presents the proposed approach. It should be noted that the results may vary depending on the selected dataset and variables. Fig 1. Proposed Method Approach

**Fig 1:** Proposed method approach.

### 2.2 Descriptive statistics

Following are the descriptive statistics of data presented in Table 1 as commutative observations. There were 1094 total observations with an average of daily new cases of around 4,595 with a standard deviation of 6,572 showing a wide variation of the daily new cases. The highest number of cases was 33,406. The average total vaccinations were approximately 49.30 million with the number of fully vaccinated people around 19.54 million. The reduction rate of the virus has been an average value of 1.04 with varying ranges of 0.51 and 2.54.

**Table 1:** Descriptive statistics.

Variable	Count	Mean	Std. Dev.	Min	25%	Median	75%	Max
**Total Cases**	1,071	1.89M	1.95M	4	20,930	867,567	4.30M	5.03M
**New Cases**	1,094	4,594.77	6,572.03	0	214	2,233	5,142	33,406
**Total Deaths**	1,020	16,866.10	16,179.13	2	347.25	10,855	35,466.25	36,853
**New Deaths**	1,094	33.69	71.45	0	1	6	29	592
**Total Vaccinations**	676	49.03M	27.21M	69	26.82M	63.36M	71.64M	72.36M
**People Vaccinated**	676	20.96M	10.33M	66	16.87M	26.09M	28.08M	28.13M
**People Fully Vaccinated**	676	19.54M	10.70M	3	9.95M	25.74M	27.39M	27.54M
**New Vaccinations**	675	107,203	139,015.66	70	8,145	39,299	158,124.5	583,111
**Reproduction Rate**	1,027	1.04	0.27	0.51	0.88	1.01	1.17	2.54

### 2.3 Data preprocessing, exploratory data analysis, and feature selection

The gathered data underwent preprocessing to ensure compatibility with the deep learning models. The preprocessing steps included:

**Data cleaning:** Eliminating any missing or inconsistent values and addressing potential outliers.

**Feature engineering:** Generating additional features, such as moving averages and growth rates, to capture relevant patterns in the data.

**Data normalization:** Scaling the features to a standard range (e.g., 0–1) to facilitate model training and convergence.

**Sequence generation:** Converting the time series data into input-output sequences with a specified window length for model training.

**Exploratory data analysis** was conducted to detect any anomalies and produce graphical visualizations.

### 2.4 Model selection, parameters, and optimization

Several Python libraries were employed, including Numpy, Matplotlib, SkLearn, Keras, Scipy, and TensorFlow. Seven advanced deep-learning models were chosen for the comparative study:

- Long Short-Term Memory (LSTM)
- Bidirectional Long Short-Term Memory (Bi-LSTM)
- Convolutional Neural Network (CNN)
- Convolutional Neural Network with Long Short-Term Memory (CNN-LSTM)
- Recurrent Neural Network (RNN)
- Gated Recurrent Network (GRU)
- Multi-layer Perceptron (MLP)

These models were selected based on their proven performance in previous SARS-COV-2 forecasting studies and their capacity to capture intricate patterns and dependencies in time series data. Further Bayesian optimization was used to select the best possible hyperparameter for the dataset for each of the algorithms and then models were evaluated again to find the best accuracy. The following are initial parameters used for each algorithm presented below in Table 2.

**Table 2:** Model parameters.

Model	Parameters
**LSTM**	• Units: 50 • Activation: relu • Optimizer: adam • Loss Function: mean_squared_error
**Bi-LSTM**	• Units: 50 • Activation: relu • Optimizer: adam • Loss Function: mean_squared_error
**CNN**	• Filters: 64 • Kernel size: 1 • Activation: relu • Pool size: 2 • Optimizer: adam • Loss Function: mean_squared_error
**CNN-LSTM**	• Filters: 64 • Kernel size: 1 • LSTM Units: 50 • Activation: relu • Optimizer: adam • Loss Function: mean_squared_error
**GRU**	• Units: 50 • Activation: relu • Optimizer: adam • Loss Function: mean_squared_error
**RNN**	• Units: 50 • Activation: relu • Optimizer: adam • Loss Function: mean_squared_error
**MLP**	• Hidden Units: Varies (10, 20, 50, 100, 200) • Activation: relu • Optimizer: adam • Loss Function: mean_squared_error

It is worth noting that each algorithm works differently with a change of parameters as per the data requirement. We have further used a batch size of 1 and trained over 100 epochs for each model. These parameters were further hyper-tuned using Bayesian optimization.

## 3. Results and discussion

We have presented first the performance of each deep learning model (LSTM, Bi-LSTM, CNN, CNN-LSTM, GRU, RNN, and MLP) without optimization and then with optimization of the models. The results are summarized using tables and graphs to illustrate the performance of the models based on various evaluation metrics (e.g., MAE, MAPE, MSE, RMSE, and R-Squared) and to visually compare their predictions with the actual data. The selected evaluation metrics were the best ones suited for time series data. However, many previous researchers have only used two metrics. However, as per previous studies, researchers just focused on one to three metrics only. Whereas the current evaluation focused on in-depth evaluation through five different evaluation metrics which were best suited for time series data.

### 3.1 Models performance metrics

Table 3 provides a summary of the evaluation metrics for each model without optimization.

**Table 3:** Model evaluation metrics without optimization.

Model	MAE	MAPE	MSE	RMSE	R^2^
LSTM	0.0064	2.404	4.412	0.0066	0.8985
Bi-LSTM	0.0078	2.374	6.361	0.0079	0.8554
CNN	0.008	2.528	8.086	0.0089	0.847
CNN-LSTM	0.0089	4.955	8.086	0.0089	0.8471
RNN	0.002	2.454	4.943	0.0022	0.9897
GRU	0.0012	2.461	1.871	0.0013	0.9961
MLP	3058.42	0.0623	18985888.755	4357.2	0.99827

#### 3.1.1 Models performance comparison without optimization

Fig 2 provides a comparison based on the actual cases in Malaysia with the predictions made by the LSTM, Bi-LSTM, CNN, CNN-LSTM, RNN, MLP, and GRU models. This visual representation allows for an intuitive understanding of each model’s forecasting accuracy.

**Fig 2:** Models’ performance without optimization.

Fig 3 provides the model’s comparison of LSTM, Bi-LSTM, CNN, and CNN-LSTM performance.

**Fig 3:** Actual vs LSTM vs Bi-LSTM vs CNN performance.

#### 3.1.2 Best-performing model without optimization

We were able to find out the best-performing model with optimization based on the evaluation metrics.

**Mean Absolute Error (MAE):** For MAE, the GRU model performs the best, with the lowest MAE (0.0012), followed by RNN (0.0020) and LSTM (0.0064). The MLP model has the highest MAE (3058.42), indicating poorer performance compared to the other models.

**Mean Absolute Percentage Error (MAPE):** The MLP model has the lowest MAPE (0.0623), followed by Bi-LSTM (2.37) and LSTM (2.40). The CNN-LSTM model has the highest MAPE (4.95596856274923), suggesting less accurate predictions compared to other models.

**Mean Squared Error (MSE):** The GRU model outperforms the other models, with the lowest MSE (1.8719), followed by the RNN (4.943) and LSTM (4.412The MLP model has the highest MSE (18985888.755), indicating a higher error rate in its predictions compared to the other models.

**Root Mean Squared Error (RMSE):** GRU model achieves the best performance with the lowest RMSE (0.0013), followed by the RNN (0.0022) and LSTM (0.0066). The MLP model has the highest RMSE (4357.27), which suggests less accurate predictions compared to the other models.

**R-squared:** MLP model has the highest R-squared value (0.9982), indicating the best performance in terms of explaining the variability in the data. The GRU model follows with an R-squared value of (0.9961), while the RNN model has an R-squared value of (0 9897). The CNN-LSTM and CNN models have lower R-squared values of (0.8471), indicating that they are less effective in explaining the variability in the data compared to the other models.

**Best Performing Model without Optimization:** Based on the above evaluation metrics and results, the GRU model consistently outperformed all other models in most of the metrics, with the lowest MAE, MSE, and RMSE values, and a high R-squared value. This indicates that the GRU model is effective in capturing the temporal dependencies in the data and providing accurate predictions for SARS-COV-2 cases in Malaysia. The RNN and LSTM models also show good performance in some metrics, but the GRU model appears to be the most effective overall.

The MLP model has the highest R-squared value, suggesting it is the best at explaining the variability in the data. However, its high MAE, MSE, and RMSE values indicate a poorer performance compared with other models. Therefore, the GRU model was the best-performing model based on the evaluation metric results for predicting SARS-COV-2 cases in this context.

#### 3.1.3 Models performance comparison with optimization

Table 4 provides a summary of the evaluation metrics for each model with optimization. For this study, we have used Bayesian optimizer for hyperparameter selection and further evaluating the model performance. We have performed minimum 10 trails to find out the best performance values for each model. The value used for optimization were ’adam’, ’sgd’, ’rmsprop’, ’nadam’, ’ftrl’, ’adagrad’, and ’adadelta’.

**Table 4:** Model evaluation metrics with optimization.

Model	MAE	MAPE	MSE	RMSE	R^2^
LSTM	0.004	2.346	3.3185	0.0005	0.9993
Bi-LSTM	0.0072	2.222	5.6419	0.0075	0.8708
CNN	0.00071	2.216	6.9800	0.0083	0.99840
CNN-LSTM	0.00042	2.1747	3.222	0.0005	0.9992
RNN	0.0039	2.1788	1.4482	0.0003	0.9996
GRU	0.0002	2.1881	1.4403	0.0003	0.9996
MLP	0.00049	2.1927	3.9551	0.0006	0.9990

Fig 4 shows the comparison of the model performance with/out optimization. The actual vs predicted values are very close to each other after optimization.

**Fig 4:** LSTM model performance comparison with/out optimization.

Fig 5 depicts a comparison of actual SARS-CoV-2 cases in Malaysia with the predictions made by the Bi-LSTM model. It shows that the model outperformed the prediction but remained close to the actual values. In comparison with the previous outcome of model evaluation without optimizer in Fig 2, the predicted values were underperforming.

**Fig 5:** Bi-directional LSTM model performance comparison with/out optimization.

Fig 6 presents the performance of the CNN model with/out optimization. It shows that the model performance has been improved after optimization. Now the predicted cases are very close to the actual cases.

**Fig 6:** CNN model performance comparison with/out optimization.

Fig 7 provides the comparison of model performance with/out optimization for CNN-LSTM model. It shows that model performance has improved after optimization.

**Fig 7:** CNN-LSTM model performance comparison with/out optimization.

Fig 8 depicts the recurrent neural network (RNN) model performance with/out optimization. It shows the improvement of model performance and now actual values are close to the predicted values.

**Fig 8:** RNN performance comparison with/out optimization.

Fig 9 shows performance of MLP model with/out optimization. It shows that model performance is almost similar to the previous performance after optimization.

**Fig 9:** MLP model performance comparison with/out optimization.

Fig 10 shows the performance of the GRU model with/out optimization. It shows that the model performance has slightly improved from the model without optimization.

**Fig 10:** GRU model performance comparison with/out optimization.

The improved performance of different models shows that optimization techniques can significantly improve performance. With adjustment of different model parameters using the learning rate, training epochs, batch sizes, and optimizer types, significantly affects the model learning from data. We will delve deeper into the analysis by comparing each evaluation metric for better understanding.

#### 3.1.4 Best performing model with optimization

We have further worked on the model for cross-validation of results by using Bayesian optimization based on the previously used metrics. The models include LSTM, Bi-LSTM, CNN, CNN-LSTM, MLP, RNN, and GRU.

**MAE:** In this case, the RNN with optimization has the lowest MAE at 0.00033, suggesting the highest prediction accuracy among the optimized models.

**MAPE:** The CNN-LSTM with optimization has the lowest MAPE at 2.1747, showing the best percentage prediction accuracy.

**MSE:** GRU with optimization has the lowest MSE at 1.4403, suggesting the best prediction accuracy in terms of squared differences.

**RMSE:** Lower RMSE values indicate better prediction accuracy. The GRU with optimization has the lowest RMSE at 0.00037, indicating the best prediction accuracy in terms of root-squared differences.

**R-squared:** The RNN with optimization has the highest R-squared value at 0.9996, indicating the best prediction accuracy in terms of the proportion of variance explained by the model.

**Summary of Best Performing Model with Optimization:** Based on the evaluation metrics, the RNN with optimization appears to be the best-performing model, as it has the lowest MAE and the highest R-squared value. The GRU with optimization also demonstrates strong performance with the lowest MSE and RMSE values.

### 3.2 Comparison between original and optimized models

When comparing the original and optimized models, we can observe improvements in the evaluation metrics for all models after optimization. Here, we present a brief comparison of each model:

**LSTM:** The optimized LSTM model shows significant improvements in all evaluation metrics, particularly in MAE (from 0.00647 to 0.00041) and R-squared (from 0.8985 to 0.9993).

**Bi-LSTM:** The optimized Bi-LSTM model exhibits slight improvements in MAPE (from 2.374 to 2.222) but otherwise, there’s not much improvement compared to the original model.

**CNN:** The optimized CNN model demonstrates significant improvements in all evaluation metrics, especially in MAE (from 0.008943 to 0.00071) and R-squared (from 0.8471953812018324 to 0.9984024271812386).

**CNN-LSTM:** The optimized CNN-LSTM model shows substantial improvements in all evaluation metrics, particularly in MAE (from 0.008943 to 0.00042) and R-squared (from 0.8471953812018324 to 0.9992621594948998).

**RNN:** The optimized RNN model exhibits significant improvements in all evaluation metrics, especially in MAE (from 0.00200 to 0.000339) and R-squared (from 0.9897 to 0.9996).

**GRU:** The optimized GRU model shows improvements in all evaluation metrics, with notable improvements in MAE (from 0.00123 to 0.000314) and R-squared (from 0.9961 to 0.99967).

**MLP:** The optimized MLP model demonstrates significant improvements in all evaluation metrics, particularly in MAE (from 3058.42 to 0.00049) and R-squared (from 0.998 to 0.9990).

In conclusion, the optimization process led to substantial improvements in the evaluation metrics for all models. The RNN and GRU models, in particular, have shown the best performance after optimization. This highlights the importance of optimizing deep learning models to achieve better prediction accuracy in forecasting tasks.

## 4. Conclusion and recommendation for future research

Future research could explore alternative feature selection and preprocessing techniques to improve model performance in the Malaysian context. The study focused on filling the research gaps by forecasting SARS-COV-2 using various deep-learning methods. The models helped to accurately forecast the changing landscape of infections in Malaysia. Additionally, our study contributes to the growing body of research on using deep learning models for pandemic forecasting, which could be applied to future public health crises. Among all tested models and based on evaluation metrics, the RNN with optimization appears to be the best-performing model, as it has the lowest MAE and the highest R-squared value. The GRU with optimization also demonstrates strong performance with the lowest MSE and RMSE values.

Additionally, studies could investigate the cause of the perfect scores observed for the RNN and MLP models and develop strategies to address these issues. Researchers could also consider applying other optimization methods other than Bayesian Optimization. By using the best-performing models to predict new cases, they can make more informed decisions about resource allocation, public health measures, and vaccination strategies.

Accurate forecasting of SARS-COV-2 dynamics is crucial for informed policy-making and resource allocation in Malaysia. Different model’s superior performance can provide valuable insights for public health officials and decision-makers in the country. By leveraging these models, authorities can better anticipate the pandemic’s trajectory, implement timely interventions, and allocate resources efficiently to mitigate the impact of the virus on the population. The discussion section highlights the performance of the deep learning models, compares the findings with previous studies, acknowledges limitations, and suggests future research directions. It also emphasizes the implications of the study’s findings for public health policy and decision-making in Malaysia.
